RETRACTED

# Long Noncoding RNA SNHG1 Activates Autophagy and Promotes Cell Invasion in Bladder Cancer

**DOI:** 10.3389/fonc.2021.660551

**Published:** 2021-05-13

**Authors:** Changcheng Guo, Xin Li, Jinbo Xie, Dan Liu, Jiang Geng, Lin Ye, Yang Yan, Xudong Yao, Ming Luo

**Affiliations:** ^1^ Department of Urology, Shanghai Tenth People’s Hospital, School of Medicine, Tongji University, Shanghai, China; ^2^ Department of Urology, Taizhou Center Hospital, Taizhou University, Zhejiang, China

**Keywords:** bladder cancer, SNHG1, autophagy, lncRNA, miRNA

## Abstract

LncRNAs play important roles in bladder cancer. However, only a few studies report on the correlation between lncRNAs expression and autophagy in bladder cancer. This study aimed to explore the effect of lncRNA on autophagy in bladder cancer. The findings showed high expression of *SNHG1* in the bladder cancer cells and tumor tissues. The high expression of *SNHG1* was positively correlated with bladder cancer cell invasion, proliferation, and autophagy. This finding implies that *SNHG1* promotes bladder cancer cell invasion and proliferation *via* autophagy. Further analysis of the mechanism of action of *SNHG1* showed that it functions as a sponge of miRNA-493 in bladder cancer. miRNA-493 binds on the 3’ -UTR of *ATG14* mRNA thus affecting ATG14 protein expression, which is implicated in autophagy. These findings are supported by previous preclinical studies using multiple Bca cell lines and TCGA, which demonstrate that *SNHG1* plays an oncogenic role by acting as a sponge of miR-493-5p or as its ceRNA. Upregulation of *SNHG1* promotes proliferation, invasion, and autophagy of bladder cancer cells through the miR-493-5p/ATG14/autophagy pathway. Therefore, *SNHG1* may act as a potential therapeutic target for the treatment of bladder cancer.

## Introduction

Bladder cancer (Bca) is the second most common malignancy of the urinary tract. There are approximately 2 million bladder cancer patients worldwide (1). Besides approximately 429,000 new cases and 165,000 deaths were reported in 2012 (2). In China, bladder cancer is the most common urologic neoplasm, with 80, 500 new cases and 32, 900 deaths reported in 2015 (3). Studies report that the incidence of bladder cancer may significantly increase in the near future due to increased exposure to risk factors such as air pollution and an increase in an aging population (4). Urothelial bladder carcinomas (UBCs) comprise more than 90% of all bladder cancer tumors and are further classified into two distinct groups: superficial non-muscle-invasive bladder cancer (NMIBC) and muscle-invasive bladder cancer (MIBC) (2, 5). Current treatment approaches are mainly effective in patients with non-metastatic bladder cancer. However, the survival rate of patients with metastatic bladder cancer is poor (6). Early diagnosis and treatment play an important role in improving the prognosis of bladder cancer. Therefore, studies should explore mechanisms underlying the malignant progression in bladder cancer for the development of effective therapies (3).

RETRACTED

Long non-coding RNAs (lncRNAs) are non-coding RNAs with more than 200 nucleotides (7). LncRNAs regulate gene expression at the post-transcriptional level, including protein synthesis, RNA maturation, and transport (8). Previous studies report that lncRNAs play a role in tumorigenesis and metastasis in different cancer types (3, 9–12). Several lncRNAs are reported to play important roles in the progression and invasion of bladder cancer. Chen et al. reported that LncRNA *LNMAT2* promotes lymphatic metastasis in bladder cancer (13). Su et al. used microarray analysis to explore the role of *FOXD2-AS1* expression in bladder cancer and found that high expression levels of *FOXD2-AS1* in bladder cancer promoted the proliferation, migration, and invasion of bladder cancer cells in both *in vitro* and *in vivo* experiments (14). Moreover, some lncRNA act as cancer-suppressor genes. Wang et al. reported that lncRNA*GAS5* promotes apoptosis in bladder cancer cells by inhibiting *EZH2* transcription (15). However, only a few studies have explored the role of lncRNAs expression in promoting autophagy in bladder cancer.

Several cancer types exhibit high expression levels of long non-coding small nucleolar RNA host genes (lnc-SNHGs). The SNHG family comprises more than 20 members, including S*NHG1, SNHG2, SNHG3, SNHG5, SNHG6, SNHG7, SNHG8, SNHG12, SNHG14* and *SNHG20*. These lncRNAs play important roles in tumor progression (16). However, the correlation between lnc-SNHGs expression and progression of bladder cancer is unknown. Therefore, in this study, we explored lnc-SNHGs expression in bladder cancer and its role in cancer proliferation and invasion.

## Materials and Methods

### BCa Samples

A total of 26 bladder cancer patients from the Department of Shanghai Tenth People’s Hospital, Tongji University (Shanghai, China) were enrolled in this study between September 2018 and June 2019. Preoperative clinical data for each patient, including age, gender, and tumor number were recorded in a computer database (**Table 1**). Bladder tumor tissues and tumor-free adjacent tissues were harvested at >2 cm from the tumor edge immediately following surgical resection in each bladder cancer patient. The specimens were divided into two groups. Tissues in one group were frozen at -80°C for use in subsequent experiments whereas tissues in the other group were preserved in 10% formaldehyde solution (62°C for 60 min) and embedded in paraffin. This study was performed following a protocol approved by the Ethics Committee of Shanghai Tenth People’s Hospital, Tongji University School of Medicine (Shanghai, China). Written informed consent for participation was obtained from each patient.

RETRACTED

**Table 1:** The associations of SNHG1 expression with clinical pathologic features in patients with bladder cancer.

Characteristics	Number	SNHG1 expression		*p* ^#^
		Low	High	
**Gender**				0.625
Male	17	9	8	
Female	9	5	4	
**Age**				0.508
≤50	11	5	6	
>50	15	7	8	
**Tumor number**				0.436
≤3	16	7	9	
>3	10	5	5	
**Histological grade**				0.817
G1	10	5	5	
G2	10	6	4	
G3	6	3	3	
**T stage**				0.154
Ta,T1	17	9	8	
T2-T4	9	4	5	
**N status**				0.097
N0	16	6	10	
N1,N2	10	4	6	
**M status**				0.756
M0	18	8	10	
M1	8	3	5	

The median expression level of SNHG1 was used as the cutoff. Patients with bladder cancer were divided into SNHG1 “Low’’ group (whose expression was lower than the median) and “High’’ group (whose expression was higher than the median).

^#^Fisher’s exact test.

### Cell Culture

Bladder cancer cells were purchased from American Type Culture Collection (ATCC, Manassas, VA). Cells were cultured in DMEM or RPMI supplemented with 10% FBS and antibiotics (100 units/mL penicillin, 100 μg/mL streptomycin) and maintained in a humidified environment containing 5% CO2 at 37°C. Lipofectamine 3000 (Invitrogen, Grand Island, NY) was used for transient transfection experiments following the manufacturer’s instructions.

### Lentivirus Packaging

pLVTHM-sh-SNHG1, psAX2 packaging plasmid, and pMD2G envelope plasmid were transfected into 293T cells using the standard calcium chloride transfection method for 48 hours to get the lentivirus soup. The lentivirus soup was collected, concentrated by density gradient centrifugation, and frozen at -80°C for further use. The sh-SNHG1 sequence and primer information is listed in the **Supplementary Table 1**.

### qPCR

Total RNAs was isolated using Trizol reagent (Invitrogen, Grand Island, NY). 1 µg of total RNA was subjected to reverse transcription using Superscript III transcriptase (Invitrogen, Grand Island, NY). Quantitative real-time PCR (qRT-PCR) was performed using a Bio-Rad CFX96 system with SYBR green to determine the mRNA expression level of the gene of interest. The expression levels were normalized using GAPDH RNA. Gene expression was calculated using modified 2^−ΔΔCt^ method, which was first described by K. Livak in PE Biosystems Sequence Detector User Bulletin 2 (17).

### Western-Blot

Cells were lysed in RIPA buffer and proteins (30 µg) were separated using 8–10% SDS/PAGE gel and transferred onto PVDF membranes (Millipore, Billerica, MA). The membranes were blocked and then incubated with appropriate dilutions of specific primary antibodies. The blots were further incubated with HRP-conjugated secondary antibodies and visualized using the ECL system (Thermo Fisher Scientific, Rochester, NY).The antibody information was as follows. Anti-LC3B antibody (ab51520,Abcam), Anti-beta Actin antibody(ab8227, Abcam), and anti-p62 antibody (ab109012, Abcam).

RETRACTED

### MTT Assay

Cell proliferation rates were determined using an MTT assay. Bladder cancer cells were seeded at 1000 per well in a 96-well plate, 24 hours after transfection with plasmids. MTT reagent was added to each well, and the plate incubated for 2 hours at 37°C. Cell proliferation assay was performed on days 1,2,3, and 4. Absorbance was measured at 450 nm before endpoint incubation. Each sample was assayed in triplicate.

### Cell Invasion Assay

Bladder cancer cells (1×105 cells) were loaded into 8μm transwells, which were pre-coated with 5-fold diluted Matrigel (BD Corning). 750μl of 10% FCS media was then placed in the lower chambers, followed by incubation at 37°C and 5% CO_2_ for 24 hours. Cells remaining in the upper chambers were removed and the membranes were fixed with methanol and stained with 0.1% (w/v) crystal violet. Invaded cells attached to the membranes were counted in ten randomly selected microscopic fields.

### Luciferase Assay

The 3’-UTR of ATG14 containing miR-493-5p responsive element was cloned into psiCHECK2 luciferase reporter vector (ATG14 wt-3’UTR). Luciferase mutant vector was obtained by mutating miR-493-5p binding site (ATG14 mut-3’UTR). Dual-Luciferase Reporter Assay System (Promega) was used to analyze the luciferase activity after transfection for 48 h.

### Immuno-Staining

Immuno-staining was performed as previously described (18). A confocal microscope was used for the visualization of the cells.

### Flow Cytometry Analysis

Cells were cultured in 6-well plates for 48 hours, and then washed and resuspended with phosphate buffer solution. After the cells were centrifugated at 300 g for 5 minutes, cells were stained with the Annexin V-FITC/PI apoptosis detecting kit (BD Biosciences, USA) for 15 minutes. A flow cytometer (BD Biosciences) was used to detect apoptosis.

### Bromodeoxyuridine (BrdU) Incorporation Assay

The cell proliferative capacity was evaluated using EdU assay kit (RiboBio, China). Approximately 10^5^ cells were seed into a 24-well plate and incubated with RPMI 1640 (10% FBS) medium for 24h. Then each well added 400μL 50μM EdU medium to incubate cells for 4 hours at 37°C. After washing the cells twice with PBS, the cells were fixed in 150μL 4% paraformaldehyde for 30 minutes, decolored with 150μL 2mg/mL glycine for 5 minutes and permeabilized in 0.5% Triton X-100 in a decolorizing shaker for 10 minutes. The cells in each well were reacted successively with 400μL 1× Apollo^®^staining solution and 400μL 1×Hoechst33342 solution for 30 minutes in the dark. Ultimately, the image of prepared cells was captured under a fluorescence microscope (Nikon, Japan) and calculated the proliferative ratio using ImageJ software.

RETRACTED

### Site-Directed Mutagenisis

Design primers according to the site to be mutated. Using KOD Plus high fidelity enzyme to perform PCR. Then the product is digested directly by adding 1ul of Dpn I to the PCR product system at 37°C for 4 hours. After PCR, inactivate the enzyme at 65°C for 10 minutes. Ultimately, amplification and sequence were performed after obtaining the ATG14 mut-3’UTR.

### Animal Studies

T24 cells transfected with the control vector (2X106) or *SNHG1* overexpression plasmid (2X106) were divided into two groups. Cells were injected into the subcutaneous layer of 6-week-old male athymic nude mice (NCI) (n = 8 mice in vector group and n=16 in *SNHG1* group). Once the tumor formation was detectable, the *SNHG1* group was divided into two groups. The 3-MA group was intraperitoneally injected with 3-MA 3 times a week for two weeks. After 6-8 weeks, mice were sacrificed, tumors excised and weighed. IVIS was used to detect tumors. A metastasis model was established by tail vein injection of T24 cells.

### Statistical Analysis

Data were expressed as mean ± SEM from at least 3 independent experiments. Statistical analyses were performed using SPSS 20.0 (SPSS Inc., Chicago, IL). P< 0.05 was considered statistically significant.

## Results

### SNHGs Is Highly Expressed in Bladder Cancer

The expression levels of *SNHG1, SNHG2, SNHG3, SNHG5, SNHG6, SNHG7, SNHG8, SNHG12, SNHG14*, and *SNHG20* were determined using qPCR.High expression levels of SNHG1 in T24 and RT4 cells were found compared with normal bladder epithelium SV-HUC1 cells (**Figure 1A**). *SNHG1* expression in T24, RT4, RT112, 253J, and DSH1 bladder cancer cells was determined and the results showed high expression levels of *SNHG1* in all the bladder cancer cells. Howerer, the highest expression levels were observed in T24 and RT4 cells compared with other cells (**Figure 1B**). Analysis of data from the TCGA database showed a positive correlation between *SNHG1* expression and overall survival. The findings indicated that high expression levels of *SNHG1* in bladder cancer patients are associated with a short survival time (**Figure 1C**). Moreover, *SNHG1* expression level is associated with the TNM stage. A high *SIHG1* expression level was observed in the N3 group whereas the pT1 stage group correlated with a low expression level. However, the *SNHG* expression levels of the clinical T stage and M stage were not significantly different (**Figures 1D–G**). A total of 26 bladder cancer patients samples from our hospital were analyzed, and the expression levels for both normal tissues and tumor tissues were determined using qPCR. The findings showed higher expression levels of *SNHG1* in tumor tissue compared with normal tissue (**Figures 1H, I**). Detailed information of the 26 bladder cancer patients is listed in **Table 1**.

RETRACTED

**Figure 1:** Long noncoding RNA *SNHG1* expression levels in bladder cancer cells and tissues. **(A)** Expression levels of *SNHG1, SNHG2, SNHG3, SNHG5, SNHG6, SNHG7, SNHG8, SNHG12, SNHG14*, and *SNHG20* in bladder cancer cell T24, RT4 and normal bladder epithelium SV-HUC1 cell; **(B)** Expression levels of *SNHG1* in T24, RT4, RT112, 253J, DSH1 bladder cancer cell and normal epithelium of bladder SV-HUC1. **(C)** Bladder cancer patients were divided into *SNHG1*-high or *SNHG1*-low groups according to the median value of *SNHG1* expression. Kaplan–Meier analysis of *SNHG1* expression and OS in bladder cancer (data from TCGA database). **(D)** *SNHG1* expression level in T-stage bladder cancer (data from TCGA database). **(E)** *SNHG1* expression level in N-stage bladder cancer (data from TCGA database). **(F)** *SNHG1* expression level in M-stage bladder cancer (data from TCGA database). **(G)** *SNHG1* expression level in pathological T-stage bladder cancer (data from TCGA database). **(H, I)** SNHG1 expression levels in tumor and normal tissues of 26 bladder cancer patients (Data presented as mean ± SD, *p < 0.05, **p < 0.01 compared to the controls).

### SNHG1 Promotes Bladder Cancer Cell Invasion and Proliferation

Cancer cells are characterized by high levels of cell proliferation and invasion. Therefore, we explored the role of *SNHG1* on bladder cancer proliferation and invasion. Overexpression *SNHG1* sequences plasmid were lentivirally transduced in T24 and RT4 cells. Both T24 and RT4 cells showed high expression of *SNHG1* after transfection (**Figure 2A**). Three different sh-sequence plasmids were used to knock down *SNHG1*. sh-*SNHG1* #1 showed higher knockdown efficiency, therefore, it was used for further experiments (**Figure 2B**). MTT proliferation assay and transwell invasion assay were used to validate the role of *SNHG1*. The findings showed that overexpression of *SNHG1* increased cell proliferation and invasion in T24 and RT4 cells. On the other hand, sh-*SNHG1* decreased cell proliferation and invasion in T24 and RT4 cells (**Figures 2C–F**). We also confirmed these results using bromodeoxyuridine (BrdU) incorporation assay (**Figure 2G**). Overexpression of *SNHG1* was found to increase cell proliferation while sh-*SNHG1* decreased cell proliferation in T24 and cells.

RETRACTED

**Figure 2:** *SNHG1* promotes bladder cancer cell proliferation and invasion. **(A)** Expression levels of *SNHG1* in T24 and RT4 bladder cancer cells. **(B)** Efficiency of the three sh-*SNHG1* sequences in T24 and RT4 bladder cancer cells. **(C)** T24 and RT4 bladder cancer cells were cultured with overexpressed *SNHG1* or control, MTT assay was used to evaluate the number of viable cells in T24 and RT4 bladder cancer cells. **(D)** T24 and RT4 bladder cancer cells were cultured with sh-*SNHG1* or control, MTT assay was used to evaluate the number of viable cells in T24 and RT4 bladder cancer cells. **(E)** T24 bladder cancer cells were cultured with overexpressed *SNHG1* or control, cell invasion assay was used to explore cell invasion of T24 bladder cancer cells. **(F)** RT4 bladder cancer cells were cultured with sh-*SNHG1* or control, cell invasion assay was used to explore cell invasion of RT4 bladder cancer cells. **(G)** T24 bladder cancer cells were cultured with sh-*SNHG1*, overexpressed *SNHG1* or control, bromodeoxyuridine (BrdU) incorporation assay was used to explore cell proliferation of T24 bladder cancer cell (Data presented as mean ± SD, *p < 0.05 compared to the controls).

### SNHG1 Promotes Bladder Cancer Cell Invasion and Proliferation Through Autophagy

To explore the mechanism of *SNHG1* in promoting bladder cancer cell invasion and proliferation, we examined autophagy in bladder cancer cells. A previous study reported that autophagy plays an important role in tumorigenesis and metastasis (19). Besides, autophagy accelerates cancer cell invasion during starvation or hypoxia (20, 21). The effect of SNHG1 on autophagy was determined using the Cyto-ID autophagy detection kit, which specifically labels autophagosomes. Overexpression of *SNHG1* significantly increased Cyto-ID fluorescence (**Figure 3A**). Further, we explored the levels of autophagy-related proteins: LC3-I, LC3-II, and P62. The results showed a significant increase in LC3-II in the *SNHG1* overexpression group, whereas P62 expression significantly decreased compared with the control group (**Figure 3B**).

**Figure 3:** SNHG1 promotes bladder cancer cell autophagy. **(A)** T24 cell was cultured with overexpressed SNHG1 or control, a Cyto-ID autophagy detection kit was used to evaluate cell autophagy. **(B)** T24 cells were cultured with overexpressed *SNHG1* or control; western-blot was used to determine the protein expression levels of LC3I, LC3II, and p62. **(C)** T24 cells were cultured with overexpressed *SNHG1*, overexpressed SNHG1 plus 5mM 3-MA, and control, MTT assay was used to evaluate the number of viable cells levels. **(D)** T24 cells were cultured with overexpressed *SNHG1*, overexpressed *SNHG1* plus 5mM 3-MA, and a control, cell invasion assay was used to determine cell invasion(Data presented as mean ± SD, *p < 0.05, **p < 0.01 compared to the controls).

RETRACTED

These findings show that *SNHG1* promotes bladder cancer cell invasion and proliferation and increases autophagy. Therefore, we investigated the mechanism of *SNHG1* in promoting bladder cancer cell invasion and proliferation. 3-Methyladenine (3-MA), an autophagy inhibitor, was found to partially or inhibit cell invasion and proliferation induced by *SNHG1* (**Figures 3C, D**). These findings implied that *SNHG1* promotes bladder cancer cell growth and invasion by inducing autophagy.

### SNHG1 Functions as a miRNA Sponge of miRNA-493 in Bladder Cancer

LncRNAs act as miRNA sponges, therefore, we explored if *SNHG1* exerted its function by interacting with tumor suppressor miRNAs in bladder cancer. Bioinformatic analysis (Diana, Starbase, Siegel lab) showed ten potential tumor suppressor miRNAs that interacted with *SNHG1*. Normalized expression levels of these potential targets in bladder cancer patients were retrieved from the GEO datasets (GSE40355) as shown in **Figure S1**. sh-*SNHG1* in T24 cells increased the expression levels of miR-195 and 493-5P (**Figure 4A**). miR-493 has been implicated in bladder cancer, therefore, we further examined explored miR-493 (**Figure S1**).

**Figure 4:** Mechanisms dissecting the role of *SNHG1* associated networks in bladder cancer autophagy. **(A)** T24 cells were cultured with sh-*SNHG1* and control, and qPCR was used to determine the expression levels of miR-182-5P, miR-23b-3P, miR-195-5P, miR-145-5P, miR-128-3P, miR-320c, miR-320a, miR-493-5P, miR-590-5P and miR-101-3P. **(B)** Binding site of *SNHG1* wild type, *SNHG1* mutation, miR-493-5P, *ATG14* 3’UTR wild type, and mutation. **(C)** qPCR was used to determine the efficiency of miR-493-5P mimics and inhibitors in T24 cells. **(D)** Treatment of T24 cells with miR-493-5P mimics or miR-493-5P inhibitor, qPCR was used to determine the relative expression level of *SNHG1* and *ATG14*. **(E)** Treatment of T24 cells with miR-493-5P mimics or control, western blot was used to determine the protein level of *ATG14*. **(F)** Luciferase assay was used to determine luciferase activity after co-transfection of *SNHG1* constructs of the wild type or mutant seed regions into T24 cells. **(G)** Luciferase assay was used to determine luciferase activity after co-transfection of *ATG* 14 3’UTR constructs of the wild type or mutant seed regions into T24 cells. **(H)** Luciferase assay was used to determine luciferase activity after co-transfection of *SNHG1* constructs of the wild type or mutant and *ATG* 14 3’UTR constructs of wild type or mutant seed regions into T24 cells (Data presented as mean ± SD, NS, no significance, *p < 0.05, **p < 0.01 compared to the controls).

RETRACTED

### The Role of SNHG1 Associated Networks in Bladder Cancer Autophagy

Further, we explored the downstream targets of the *SNHG1*/miRNAs axis using bioinformatic tools (Targetscan, Starbase, MicroRNA.org) and literature search. The focus was on ATG14, an autophagy-related protein whose 3’UTR is a potential of miR-493. Binding site information of SNHG1/miRNAs/ATG14 is shown in Fig4B. The efficacy of miR-493-5p mimics and inhibitor was explored (**Figure 4C**). Besides, *SNHG1* and *ATG14* expression levels were determined by qPCR. The results showed that miR-493-5p significantly reduced the mRNA expression levels of *SNHG1* and *ATG14*. On the other hand, the addition of miR-493-5p inhibitor significantly increased the expression levels of *SNHG1* and *ATG14* (**Figure 4D**). Moreover, miR-493-5p decreased the expression of ATG14 protein (**Figure 4E**). Based on the predicted position, we mutated SNHG1 using site-directed mutagenesis and determined the effect using luciferase assay. The results revealed that miR-493-5p changed wild-type *SNHG1* luciferase activity compared with the group lacking the SNHG1 mutation (**Figure 4F**). Furthermore, we mutated *ATG14* 3’UTR and observed that miR-493-5p significantly changed *ATG14* 3’UTR wild type luciferase activity, compared with the group lacking the *ATG14* 3’UTR mutation, which showed no activity (**Figure 4G**).

Analysis of the mechanisms underlying the miR-493-5p and *ATG14* expression levels revealed potential binding sites located on the 3’ -UTR of *ATG14* mRNA (**Figure 4B**). A reporter assay with psiCheck2 vector carrying wild-type and mutant miRNA target sites was used for further analysis. The results showed that miR-493-5p suppressed luciferase activity in T24 cells with wild-type *ATG14* 3’UTR. However, miR-493-5p did not affect on luciferase activity in mutant *ATG14* 3’UTR (**Figure 4H**). Suppression of luciferase activity was reversed with the addition of wild-type *SNHG1* (**Figure 4H**). These findings imply that *SNHG1* suppresses *ATG14* 3’-UTR protein expression by binding to miR-493-5p.

### miR-493-5p Modulates SNHG1 Induced Invasion and Autophagy in Bladder Cancer Cells

To further explore the role of miR-493-5p in SNHG1 mediated invasion and autophagy in bladder cancer cells, we evaluated T24 cell invasion *via* overexpression of miR-493-5p. The results showed that miR-493-5p suppressed T24 cell invasion (**Figure 5A**) and that overexpression of *SNHG1* in T24 cells correlated with high T24 cell invasion ability. However, the increased invasion ability was reversed by overexpression of miR-493-5p (**Figure 5B**). Besodes, 3-Methyladenine (3-MA), an autophagy inhibitor, partially or totally inhibited cell invasion and proliferation induced by *SNHG1*(**Figure 5B**). Immunofluorescence and confocal analysis showed that *SNHG1* increased the level of LC3, an important marker of autophagy, whereas miR-493-5p overexpression inhibited LC3 expression (**Figure 5C**). Further, we determined the protein levels of LC3-I, LC3-II, and P62 which are associated with autophagy. The results showed that miR-493-5p inhibited the increased levels of LC3-II mediated by *SNHG1*, whereas P62 was highly expressed (**Figure 5D**). These results imply that *SNHG1* promotes T24 cell invasion and autophagy through miR-493-5p.

RETRACTED

**Figure 5:** miR-493-5p plays an important role in *SNHG1* induced bladder cell invasion and autophagy. **(A)** T24 bladder cancer cells were cultured with miR-493-5P mimics, cell invasion assay was used to evaluate the cell invasion ability of T24 bladder cancer cells. **(B)** T24 bladder cancer cells were cultured with *SNHG1* and *SNHG1* plus miR-493-5P mimics, cell invasion assay was used to evaluate cell invasion ability of T24 bladder cancer cells (UP); 24 bladder cancer cells were cultured with *SNHG1* and *SNHG1* plus miR-493-5P mimics with or without 3-MA, cell invasion assay was used to evaluate cell invasion ability of T24 bladder cancer cells (down) **(C)** T24 cells were cultured with overexpressed *SNHG1* or control or *SNHG1* plus miR-493-5P, Cyto-ID autophagy detection kit was used to evaluate cell autophagy. **(D)** T24 cells were cultured with overexpressed *SNHG1* or control or *SNHG1* plus miR-493-5P; western-blot was used to determine the protein expression levels of LC3I, LC3II and p62 (Data presented as mean ± SD, *p < 0.05, **p < 0.01 compared to the controls).

### SNHG1 Promotes Bladder Cancer Cell Proliferation *In Vivo*

To further examine the biological functions of *SNHG1 in vivo*, T24 cells transfected with a control vector or *SNHG1* overexpression plasmid were inoculated into nude mice. Further analysis demonstrated that *SNHG1* overexpression increased tumor volume and weight (**Figures 6A, B**). However, the addition of 3-MA (25mg/kg) significantly reduced *SNHG1* induced tumor volume and weight (**Figures 6A–D**). IHC staining results also showed that *SNHG1* promotes bladder cancer cell proliferation *via* autophagy, and these findings were consistent with the *in vitro* findings (**Figure 6E**).

RETRACTED

**Figure 6:** T24 cells stably transfected with *SHNG1* plasmid or vector were injected subcutaneously into nude mice to establish subcutaneous xenograft tumors (5 × 106 cells per mice, each group contains 8 mice). Tumor growth curve and weight decreased in the *SNHG1* group compared with the vector group. Data are presented as mean ± SEM, **P < 0.01 versus vector group. **(A)** After sacrificing the mice, the tumor tissues were obtained. **(B)** The tumor volume was measured at different times; **(C)** IVIS imaging was used to determine the tumor size in different groups **(D)** The quantitative analysis of IVIS imaging in different groups **(E)** The IHC detection of LC3-I, LC3-II, and P62 in subcutaneous xenografts of the three groups. (Data presented as mean ± SD, **p<0.01 compared to the controls).

Therefore, *SNHG1* promotes T24 cell proliferation whereas 3-MA inhibits miR-493-5p/ATG14/autophagy pathway *in vivo*.

## Discussion

Bladder cancer (Bca) is the second most common malignancy of the urinary tract. Currently, TURBt and cystectomy are the conventional treatment approaches for non-metastatic bladder cancer, with acceptable efficacy. However, the survival of patients with metastatic bladder cancer is poor (6), hence the need to explore new therapies for metastatic bladder cancer. Previous studies report that aberrantly expressed lncRNAs play important roles in tumorigenesis and can be used to predict patient survival outcomes. However, the relationship between lncRNAs and Bca tumorigenesis has not been fully elucidated.

To the best of our knowledge, this study for the first time explores the expression of *SNHG1* in Bca tissue and cell lines. The findings show that high levels of *SNHG1* correlate with the poor prognosis of Bca patients. The results further showed that high expression of *SNHG1* in Bca promotes Bca cell proliferation and invasion *in vitro* and increases autophagy. *SNHG1* mainly exerted its effect on Bca by directly targeting miR-493-5p. To validate these results, we further investigated the miR-493-5p tumor suppressor function. The results showed that transfection of miR-inhibitor reverses the si-SNHG1 tumor-suppressive effect on Bca cell growth and invasion. These findings indicate that *SNHG1* and miR-493-5p modulate tumor progression in Bca through synergistic activity. Moreover, overexpression of *SNHG1* can be a potent oncogenic marker in Bca, therefore, it can be used as a potential novel therapeutic target in renal cancer. Analysis of data retrieved from the TCGA database showed that high levels of *SNHG1* were positively correlated with the poor prognosis of Bca patients. Further analysis showed a high expression level of *SNHG1* in the N3 group and low expression in the pT1 stage group. However, the expression levels of *SNHG1* in the clinical T stage and M stage were not significantly different. This finding was attributed to the limited number of Bca patients in the TCGA database.

RETRACTED

LncRNAs are noncoding transcripts comprising more than 200 nucleotides. LncRNA is a large and significantly diverse RNA family. lncRNAs induce chromatin modifications, mediate gene silencing, and act as guide molecules and scaffolds for proteins resulting in the formation of cellular substructures. In addition, they control protein synthesis, RNA maturation and transport (22–24). LncRNAs also play a sponge role, competing with other genes for miRNA binding and modulate the regulatory effect of miRNAs on targeted mRNAs (25, 26). This posttranscriptional mechanism alters the components of the endogenous regulatory interaction networks. Notably, ncRNAs sharing miRNA recognition element with mRNAs can act as miRNA decoys and participate in “competing endogenous RNA” (ceRNA) activity (27, 28). A previous study reported that ceRNA plays an important role in cancer. In pancreatic cancer, *NORAD* functions as a ceRNA to regulate the expression of the small GTP binding protein, RhoA by competing for hsa-miR-125a-3p, thus promoting EMT (29). In gallbladder cancer, lncRNA-*PAGBC* competitively binds to the tumor-suppressive microRNAs, miR-133b and miR-511 to promote tumor growth and metastasis and to activate the *AKT/mTOR* pathway (30). In renal cell carcinoma, HOTAIR functions as a ceRNA for miR-217 to facilitate *HIF-1α* expression and upregulates AXL level promoting renal cell carcinoma proliferation, migration, and EMT process, and inhibiting apoptosis (31). In prostate cancer, lncRNA-ROR significantly increases the levels of miR-145 in *CD44+/CD133+* human prostate cancer stem cells. MiR-145 prevents cell proliferation by decreasing *Oct4* expression.

Based on these findings, we explored the relationship between ceRNA and *SNHG1* in bladder cancer. The findings showed that *SNHG1* functions as a ceRNA of miR-493-5p. Interestingly, we also found that miR-493-5p significantly decreased the mRNA expression of *SNHG1*, while the addition of a miR-493-5p inhibitor significantly increased expression the *SNHG1* expression levels. The reason for this maybe that *SNHG1* is also the target gene of miR-129-5P. We further confirmed that miR-493-5p plays an important role in *SNHG1* induced bladder cell invasion and autophagy. Data were retrieved from the GEO database and used to investigate the expression of miR-493-5p in bladder cancer cells. The results showed low expression levels of miR-493-5p in bladder cancer, and that miR-493-5p was associated with autophagy. Moreover, miRNA-493 was found to modulate *ATG14* mRNA levels and ATG14 protein expression levels by binding to the 3’ -UTR of *ATG14*, a protein implicated in mediating autophagy.

RETRACTED

## Conclusion

The findings of this study show that *SNHG1* plays an oncogenic role by sponging miR-493-5p or acting as its ceRNA. Besides, high expression of *SNHG1* promotes proliferation, invasion, and autophagy of bladder cancer cells *via* the miR-493-5p/ATG14/autophagy pathway. These findings imply that the *SNHG1* is a potential therapeutic target for the treatment of bladder cancer.

## Data Availability Statement

The datasets presented in this study can be found in online repositories. The names of the repository/repositories and accession number(s) can be found in the article/**Supplementary Material**.

## Ethics Statement

The studies involving human participants were reviewed and approved by Shanghai Tenth People’s Hospital, Tongji University. The patients/participants provided their written informed consent to participate in this study. The animal study was reviewed and approved by Shanghai Tenth People’s Hospital, Tongji University. Written informed consent was obtained from the owners for the participation of their animals in this study.

## Author Contributions

CG designed the experiments, performed experiments, analyzed the data and wrote the paper. XL initiated the study, designed the experiments and wrote the paper. DL provided Bca samples. JG performed experiments. LY and YY did the animal study, XY and ML initiated the study, designed the study and wrote the paper. JX performed experiments. All authors contributed to the article and approved the submitted version.

## Funding

This study was funded by the National Natural Science Foundation of China (81802518) and the Shanghai Science and Technology Commission Foundation (17ZR1421800).

## Conflict of Interest

The authors declare that the research was conducted in the absence of any commercial or financial relationships that could be construed as a potential conflict of interest.

## Supplementary Material

Supplementary Figure 1
**(A–I)** Normalized expression level of potential miR-RNA targets in bladder cancer patients retrieved from the GEO datasets (GSE40355). **(J)** T24 cells were cultured with 5mM DMSO or 5mM 3-MA, MTT assay was used to evaluate cell proliferation levels.

RETRACTED

Supplementary Figure 2 T24 bladder cancer cells were cultured with overexpressed SNHG1 or knocking down SNHG1, and the cells were seeded at a density of 4 x 105 cells/well. After 12 h post-treatment, cells were stained with annexin V and propidium iodide and subjected to flow cytometric analysis. The result is representative of three independent experiments.

Supplementary Table 1 Primer information.
